# Effect of New Nursing Team Management Mode on Self-Efficacy, Compliance, and Quality of Life of Patients with Chronic Kidney Disease and Its Chain Mediating Effect

This article has been retracted.

**DOI:** 10.1155/2022/2071893

**Published:** 2022-07-05

**Authors:** Jie Zheng, YueJuan Jing, AoHan Guo, ShuYan Wu, Rong Liu, LinJun Zhai

**Affiliations:** ^1^Nursing College, Shanxi Medical University, Taiyuan 030001, China; ^2^Hemodialysis Room, The Second Hospital of Shanxi Medicine University, Taiyuan 030001, China

## Abstract

Chronic kidney disease (CKD) is one of the serious diseases that lead to a series of metabolic disorders, and its process is irreversible. In order to explore the intervention effect of the new nursing team intervention program in patients with CKD, 100 patients with CKD from May 2020 to May 2021 were randomly selected in this paper and divided into the traditional group and the combined group. The comparison of clinical nursing shows that the new nursing team management model improves the compliance, self-management efficiency, and quality of life of patients with CKD, which is worth recommending in nursing practice.

## 1. Introduction

CKD patients have progressive deterioration of renal function, which leads to a series of metabolic disorders. This process is irreversible. At present, no effective treatment has been developed clinically. Maintenance hemodialysis (MHD) is often used to maintain life [1]. Most chronic renal failure (CRF) patients have psychological problems of varying degrees, resulting in a low quality of life [2]. Compliance and self-efficacy are the main factors affecting the therapeutic effect of MHD, so improving treatment compliance and self-efficacy is of great significance to reduce the negative emotions and improve the quality of life of MHD patients with chronic renal failure [3]. Team nursing is an emerging nursing intervention mode in recent years. By optimizing professional intergroup nursing teams, patients can be provided with higher quality nursing services, thus improving the treatment enthusiasm, self-efficacy, and mobility of patients, helping to improve the quality of life of patients, and achieving certain achievements in the field of chronic disease care [4]. At present, there are few literature on the application of the team effect in patients with CKD. Therefore, this study applied new team nursing to patients with CKD to further observe the influence of new team interaction on medication compliance, self-efficacy, and quality of life of patients with CKD as well as the chain mediating effect of various scores, providing theoretical support for subsequent studies.

The rest of this paper is organized as follows: Section 2 discusses related work, followed by the methods of clinical diagnosis and data statistics in Section 3. The case analysis and comparison are discussed in Section 4.  Section 5 concludes the paper with a summary and future research directions.

## 2. Related Work

The incidence of end-stage renal disease is increasing year by year, and maintenance hemodialysis plays an important role in the care of patients with end-stage renal disease. Long-term hemodialysis treatment will cause complications such as abnormal blood pressure, malnutrition, and metabolic disorders, aggravating the psychological burden of patients [5].

The results of this study showed that patients in the combined group had a higher nursing improvement effect in self-efficacy, quality of life and medication mobility, suggesting that the application of professional nursing team management intervention can further improve the nursing effect of patients. This paper analyzes the reasons for implementing management intervention, and then effectively adjusts the nursing plan. At the same time, the influence of artificial nursing method factor deviation on nursing effect should be solved. In addition, with specialist physicians, the nursing focus can be arranged by doctors, which can further optimize the nursing intervention process for patients. Meanwhile, nursing management programs such as psychological counseling can focus on cultivating and improving the self-management efficiency of patients, and all kinds of nursing measures are conducive to improving the treatment compliance of patients [6]. Studies have shown that lower self-efficacy level will indirectly lead to a lower quality of life, and improving self-efficacy levels can effectively improve patients' quality of life [7, 8].

The other paper concludes that patient self-efficacy is a good factor to predict patient compliance through multiple regression model analysis, and the higher the self-efficacy, the better the patient compliance [9]. The paper by Hamerman shows that enhancing self-efficacy could effectively improve patients' compliance and thus indirectly improve patients' quality of life [10]. The results of this study show that compliance is positively correlated with self-efficacy and quality of life, while self-efficacy is positively correlated with quality of life, and compliance has a chain mediating effect between self-efficacy and quality of life in elderly patients with arteriosclerotic occlusive disease. Analysis of the reasons is perhaps the good compliance of patients with high self-discipline. Although the quality of life is affected by many factors such as environment, psychological, and disease severity, the key factors influencing the quality of life, the patient's compliance plays a decisive role in patients with disease severity. Good adherence can greatly improve the clinical curative effect. Thus, the severity of the disease can be effectively reduced and the quality of life can be improved [11]. Increased self-efficacy of patients promotes the increase in self-care behaviors of patients and effectively improves their physical and mental symptoms. Improving the self-efficacy of patients can assist patients in comprehensively controlling clinical symptoms and achieve the clinical purpose of improving quality of life [12]. Self-efficacy is the main predictor of maintaining and changing patients' medication compliance. Good self-efficacy of patients indicates that they can effectively control psychological stress and comprehensive efficacy, so they are more confident in adherence to medication treatment and thus improve patients' medication compliance and clinical efficacy.

Compliance plays a chain mediating role between self-efficacy and quality of life, possibly because the improvement of self-efficacy and compliance can improve the quality of life of patients, while self-efficacy can indirectly improve the quality of life of patients through the improvement of compliance. There are still some shortcomings in this study, such as a small sample size and incomplete observation indexes. Therefore, the sample size and observation indexes should be increased in subsequent studies to conduct in-depth studies with large samples and multicenters.

## 3. Clinical Treatment Methods and Evaluation Indicators

### 3.1. Patients and Treatment

A total of 100 patients with CKD who received maintenance hemodialysis treatment in our hospital from May 2020 to May 2021 were selected for the study. They are divided into the traditional group and the combined group according to the random number table method, with 50 patients in each group. There are 39 males and 11 females aged 40–60 years in the joint group, with an average of (51.27 ± 2.23) years. Body mass index (BMI) is 18–27 kg/m^2^, with an average of (23.34 ± 2.83) kg/m^2^. The mean dialysis time is (5.98 ± 1.48) months. There are 38 males and 12 females aged from 41 to 63 years in the traditional group, with a mean of (51.33 ± 2.19) years. BMI ranged from 18 to 27 kg/m^2^, with a mean of (23.31 ± 2.9) kg/m^2^, and dialysis lasted 4–6 months, with a mean of (5.97 ± 1.43) months (*P* > 0.05), with comparability.

The inclusion criteria include the following aspects: (1) meeting CKD diagnostic criteria and confirmed by laboratory examination; (2) normal communication and feedback; (3) receiving dialysis treatment for more than 3 months; (4) complete clinical data; and (5) this is the first visit to the hospital [13, 14].

The exclusion criteria include the following aspects: (1) pregnancy and lactation; (2) kidney transplant recipients; (3) a history of mental illness or communication disorder; (4) organic cardiovascular and cerebrovascular diseases; and (5) receiving other sports and psychological intervention during the study.

The traditional group adopts routine nursing, including adjusting indoor temperature and humidity, ensuring a quiet environment in the ward and examination room, regular ventilation, distributing disease brochures to patients, answering questions raised by patients on time, and visiting wards on time. On the basis of conventional nursing in the traditional group, the combined group applied the new nursing team management mode to intervene, constructed a nursing team management group, and assigned special nursing tasks and corresponding patients to each group, according to the frequency of nursing 3 times a week, 40 min each time. The specific work is divided into the following steps: (1) explain the intervention process and related matters needing attention to patients and their families in detail, explain the pathogenesis and diagnosis process in the form of PPT, short videos, pictures and books, and guide patients to introduce their personal diagnosis and treatment experience through symposia; (2) specialists carry out personalized medication and diet nursing programs according to the psychological and behavioral changes of patients, patiently explain relevant matters for attention and guide the patient's family members to participate in patient care; and (3) guide patients to face negative emotions, adjust treatment mentality, make patients face the disease and actively cooperate with treatment, and organize patients to summarize experience regularly. The subjects are followed up for 6 months, and the 4 observation time points are respectively before the nursing intervention, 1, 3, and 6 months after nursing intervention and marked as T1-T4.

### 3.2. Observation Indicators

The observation indicators are divided into the following steps: (1) General Self-efficacy Scale (GSES) is used at all 4 time points to evaluate the patients' self-efficacy. The full score was 40, and self-efficacy increased with the increase of the score; (2) the patient's adherence is evaluated according to the Morisky Medication Adherence Scale (MMAS-8) [15]. The first seven adherence items all contain yes and no, each of which is scored in accordance with 0∼1 points. The eighth item is divided into five items according to the frequency of occurrence and is marked as 1 point, 0.75-point, 0.5-point, 0.25 point, and 0 point from low to high. The total score is 0–8, and the medication compliance increased with the increase of the score; (3) the WHO Quality of Life-100 (WQL-100) scale is used to evaluate the quality of life of patients at 4 time points [16]. There are 25 items in total, including three dimensions of independence, psychology, and life comfort, according to the 5-level scoring system. The total score is 25–125, and the quality of life increases with the increase in the score.

### 3.3. Statistical Methods

The SPSS 24.0 software is used to process the data in the study. The counting data is represented by the *χ*^*2*^ test, the measurement data is represented by the *t*-test, and the mean ± standard deviation (‾*x* ± *s*), and the multiple groups of data are represented by the *F* test. The Mauchly test is used to compare the data at different time points within the group. *P* > 0.05 indicated that the covariance matrix is full of football symmetry. The sequential inspection method is used to test the chain mediation effect of compliance between self-efficacy and quality of life.

## 4. The Case Analysis and Comparison

### 4.1. Comparison of Self-Efficacy at Four Research Time Points

The self-efficacy level of the two groups has an increasing trend, and the T2-T4 self-efficacy scores of the combined group are higher than those of the traditional group, with statistical significance (*P* < 0.05), as shown in Table 1.

In Figure 1, a, b, c, and d are given as comparison with other time points (*P* < 0.05). ^#^ is compared with the traditional group (*P* < 0.05).

### 4.2. Comparison of Compliance at Four Study Time Points

The compliance level of the two groups shows an increasing trend, and the T2-T4 compliance score of the combined group is higher than that of the traditional group, with statistical significance (*P* < 0.05), as shown in Table 2.

In Figure 2, a, b, c, and d are given as comparison with other time points (*P* < 0.05). ^#^ is compared with the traditional group (*P* < 0.05).

### 4.3. Comparison of Quality of Life at Four Research Time Points

The quality of life of the two groups shows an increasing trend, and the scores of T2-T4 independence, psychological, and life comfort in the combined group are higher than those in the traditional group, with statistical significance (*P* < 0.05), as shown in Table 3.

In Figure 3, a, b, c, and d are given as comparison with other time points (*P* < 0.05). ^#^ is compared with the traditional group (*P* < 0.05).

### 4.4. Chain Mediating Effect of Compliance on Self-Efficacy and Quality of Life in Patients with CKD

According to the mediation effect testing procedure proposed in the literature, the mediation effect should satisfy two conditions: (1) the independent variable affects the mediation variable, the dependent variable and the mediation variable can affect the dependent variable; and (2) taking self-efficacy and compliance as independent variables and mediating variables, and quality of life as the dependent variable, step regression analysis is conducted to clarify the impact of compliance and self-efficacy on quality of life. The results show that both compliance and self-efficacy could affect the quality of life. In Table 4, “-” means a blank item (^a^*P*＜0.05).

Taking self-efficacy as an independent variable and compliance as a dependent variable, stepwise regression analysis was conducted to clarify the influence of self-efficacy on compliance, and the results show that self-efficacy could affect compliance, as shown in Table 5. Therefore, compliance is a mediating variable between self-efficacy and quality of life, and compliance can play a chain mediating role between self-efficacy and quality of life. In Table 5, “-” means a blank item (^a^*P*＜0.05).

The bootstrap method is used to further test the significance of each pathway, and the results show that the chain mediation effect from compliance to quality of life has a 95% CI of 0.031–0.162. If 0 is not included in the interval, the mediation effect is significant, as shown in Table 6.

## 5. Conclusions

In conclusion, the intervention of CKD patients with the new nursing team management model can achieve good clinical effects. The combined program can help improve self-efficacy and medication compliance and play a positive role in improving patients' quality of life, which is worthy of clinical promotion.

## Figures and Tables

**Figure 1:** Changes in the self-efficacy score across the four study time points.

**Figure 2:** Changes in adherence scores across the four study time points.

**Figure 3:** Changes in quality of life at different time points: (a) the stand-alone capability; (b) the psychology; (c) the life comfort.

**Table 1:** Demographic and baseline clinical characteristics of patients.

Group	Time point	Self-efficacy score
Joint group (*n* = 50)	T1	10.23 ± 1.01
	T2	19.63 ± 1.12
	T3	27.43 ± 1.25
	T4	37.55 ± 2.02

Traditional group (*n* = 50)		
	T1	10.19 ± 1.21
	T2	16.43 ± 1.02
	T3	24.43 ± 1.15
	T4	32.55 ± 1.62

*F*_time point_		455.768
*P*_time point_		<0.001
*F*_point_^*∗*^_group_		517.105
*P*_point_^*∗*^_group_		<0.001

**Table 2:** Comparison of adherence across the four study time points (‾*x* ± *s*).

Group	Time point	Compliance score
Joint group (*n* = 50)	T1	2.23 ± 0.11
	T2	3.63 ± 0.22
	T3	5.43 ± 0.35
	T4	6.55 ± 0.62

Traditional group (*n* = 50)		
	T1	2.21 ± 0.10
	T2	3.23 ± 0.15
	T3	4.12 ± 0.22
	T4	5.25 ± 0.37

*F*_time point_		434.548
*P*_time point_		<0.001
*F*_point_^*∗*^_group_		522.143
*P*_point_^*∗*^_group_		<0.001

**Table 3:** Changes in quality of life at different time points (‾*x* ± *s*).

Group	Time point	Stand-alone capability	Psychology	Life comfort
Joint group (*n* = 50)	T1	9.12 ± 1.01	20.23 ± 1.01	9.33 ± 1.01
	T2	18.52 ± 1.11	49.63 ± 3.12	19.63 ± 1.14
	T3	26.31 ± 1.24	57.43 ± 5.25	24.43 ± 1.23
	T4	36.44 ± 2.04	77.55 ± 6.02	32.55 ± 1.32

Traditional group (*n* = 50)				
	T1	9.09 ± 1.11	20.19 ± 1.21	9.23 ± 1.01
	T2	15.23 ± 1.24	36.43 ± 3.02	14.63 ± 1.12
	T3	21.33 ± 1.23	44.43 ± 4.15	19.43 ± 1.17
	T4	30.45 ± 1.55	62.55 ± 5.62	24.55 ± 1.21

*F*_time point_		455.768	325.438	295.548
*P*_time point_		<0.001	<0.001	<0.001
*F*_point_^*∗*^_group_		517.105	477.122	647.335
*P*_point_^*∗*^_group_		<0.001	<0.001	<0.001

**Table 4:** Quality of life model test of CKD patients.

Project self-efficacy	First steps		Second step		Third step	
	*β*	*t*	*β*	*t*	*β*	*t*
Compliance	—	—	-0.239	8.003a	-0.224	7.625_a_
Project	—	—	—	—	-0.388	8.749_a_
*F*	80.157		76.473		87.447	
*R* ^*2*^	0.50		0.54		0.61	
P	＜0.001		＜0.001		＜0.001	

**Table 5:** Model test of adherence in CKD patients.

Project	First steps		Second step		Third step	
	Β	*t*	*β*	*t*	*β*	*t*
Self-efficacy	—	—	—	—	-0.390	8.751_a_
*F*	80.155		76.472		87.443	
*R* ^*2*^	0.52		0.55		0.62	
P	＜0.001		＜0.001		＜0.001	

**Table 6:** Path and effect decomposition of self-efficacy on quality of life.

Effect	Path relationship	Effect value	Effect quantity
Direct effect	Compliance ⟶ quality of life	-0.389	64.59
Mesomeric effect	Self-efficacy⟶ compliance ⟶ quality of life	-0.100	16.72
Total mediation effect	—	-0.210	35.31
Gross effect	—	-0.601	100.00

## Data Availability

The simulation experiment data used to support the findings of this study are available from the corresponding author upon request.

## References

[1] Du L., Zu M. (2018). Effects of individualized dietary guidance on nutritional status, calcium and phosphorus metabolism and blood glucose management in patients with chronic renal failure on maintenance hemodialysis. *Anhui pharmaceutical*.

[2] Adamczak M., Surma S. (2021). Metabolic acidosis in patients with CKD: epidemiology, pathogenesis, and treatment. *Kidney Disease*.

[3] Asadipooya K., Abdalbary M., Ahmad Y., Kakani E., Monier-Faugere M.-C., El-Husseini A. (2021). Bone quality in CKD patients: current concepts and future directions - Part I. *Kidney Disease*.

[4] Oliverio A. L., Bramham K., Hladunewich M. A. (2021). Pregnancy and CKD: advances in care and the legacy of dr susan hou. *American Journal of Kidney Diseases*.

[5] Calvani M., Benatti P., Mancinelli A. (2019). Effects of l-carnitine on the nutritional status and cardiac function of patients with maintenance hemodialysis and end-stage renal disease. *Clinical misdiagnosis and mismanagement*.

[6] Gao G., Zhang P., Xu B. (2022). Analysis of bioelectrical impedance spectrum for elbow stiffness based on hilbert-huang transform. *Contrast Media and Molecular Imaging*.

[7] Chen Q., Qu S., Huang X. (2019). Reliability and validity analysis of mMAS-8 in the evaluation of medication compliance in patients with chronic cardiovascular disease. *Chinese pharmacy*.

[8] Ferreira J. P. (2020). Health‐related quality of life scores: ending the minimum 5‐point difference as the clinically meaningful threshold. *European Journal of Heart Failure*.

[9] Chen J., Chiang C. (2021). Uremic toxins and protein-bound therapeutics in AKI and CKD: up-to-date evidence. *Toxins*.

[10] Wang L., Shan M. (2021). Effects of empathy nursing on the quality of life and treatment compliance of elderly patients with cerebral infarction. *American Journal of Tourism Research*.

[11] Young C. A., Mills R., Rog D. (2021). Quality of life in multiple sclerosis is dominated by fatigue, disability and self-efficacy. *Journal of the Neurological Sciences*.

[12] Riazi H., Madankan F., Azin S. A., Nasiri M., Montazeri A. (2021). Sexual quality of life and sexual self-efficacy among women during reproductive-menopausal transition stages and postmenopause: a comparative study. *Women’s midlife health*.

[13] Gao G., Cao L., Du X. (2022). Comparison of minimally invasive surgery transforaminal lumbar interbody fusion and TLIF for treatment of lumbar spine stenosis. *Journal of Healthcare Engineering*.

[14] Hamerman E. J., Aggarwal A., Poupis L. M. (2021). Generalized self-efficacy and compliance with health behaviours related to COVID-19 in the US. *Psychology and Health*.

[15] Anaforoglu I., Sancak S., Akbas E. M. (2021). Effects of treatment adherence on quality of life in hypoparathyroid patients. *Experimental and Clinical Endocrinology & Diabetes*.

[16] Tabernero C., Caprara G. V., Gutiérrez-Domingo T. (2021). Positivity and self-efficacy beliefs explaining health-related quality of life in cardiovascular patients. *Psicothema*.

